# Preservation of Autologous Brachiocephalic Vessels with Assistance of Three-Dimensional Printing Based on Convolutional Neural Networks

**DOI:** 10.1155/2022/6499461

**Published:** 2022-03-17

**Authors:** Yu Yan, Yan-Yan Su, Zhong-Ya Yan

**Affiliations:** ^1^Department of Cardiovascular Surgery, The Second Affiliated Hospital of Anhui Medical University, Hefei, China; ^2^Department of Anatomy, Anhui Medical University, Hefei, China

## Abstract

**Background:**

Preservation of autologous brachiocephalic vessels in Stanford type A aortic dissection has good short-time outcomes. However, getting access to the details is not easy by conventional examination methods. This study is aimed at reconstructing the aortic arch model by three-dimensional (3D) printing based on convolutional neural networks (CNN) to understand the details for performing surgery.

**Methods:**

Three patients with type A aortic dissection from October 2017 to June 2018 were indicated for simplified Sun's procedure. Convolutional neural network (CNN) is used as a deep learning model, and the model was preset by transfer learning. The genetic algorithm (GA) was used to optimize the parameters. The aortic arch models were reconstructed using the segmented image.

**Results:**

The predicted damage area (mean 0.021 mm^2^) of the model optimized by deep learning was consistent with the experimental results (mean 0.023 mm^2^). Among the three patients, one patient died due to multiple organ failure and septic shock on the 11th day after surgery. The other two patients were cured, no reoperation was reported, and their cardiac functions were defined as class I during the 13 and 20 months of follow-up.

**Conclusion:**

It is feasible to use CNN to optimize the manufacturing of the aortic arch models.

## 1. Introduction

Stanford type A aortic dissection is a life-threatening disease that deteriorates rapidly. The incidence of this disease has been increasing in China [1]. Without medical intervention, the mortality rate of this disease increases by 1% each hour after its onset and reaches 30-50% within 48 hours [2, 3]. At present, Stanford type A aortic dissection is mainly treated by surgery. Among different surgical procedures, Sun's procedure (total aortic arch replacement combined with stented elephant trunk implantation) [4] applies to a variety of patients with complex changes in aortic arch morphology [5].

Although well accepted, this procedure is complicated because of its multiple anastomose. The autologous brachiocephalic vessel preserved Sun's procedure is one of the simplified procedures of conventional Sun's procedure, and it has excellent shot-term outcomes [6, 7]. Considering the requirement of comprehensive understanding of the details of patients' aortic arch (including the autologous brachiocephalic vessels) for applying the simplified procedure and the complex morphology of the aortic arch itself, the information obtained from conventional imaging examination before surgeries are relatively limited [8].

Convolutional neural networks (CNN) predictive analysis has been widely used in biomedical field [9–11]. Based on the patients' computed tomography angiography (CTA) data, we tried to reconstruct the aortic arch models using three-dimensional (3D) printing technology based on the CNN to make an accurate diagnosis and grasp the strict surgical indications of this simplified procedure properly.

## 2. Material and Methods

### 2.1. Case Information

From October 2017 to June 2018, there were three patients with type A aortic dissection who were indicated for simplified Sun's procedure, and the clinical data of patients are listed in Table 1.

### 2.2. Experimental Data Set

CT scan images of patients were selected with scanning thickness of 3.0 mm and reconstruction resolution of 512 × 512. Aortic CTA was performed, and the occurrence of type A aortic dissection was confirmed in each patient. First, we transformed the original CTA data into a rough 3D graphic of the aortic lumen, using 3D image processing software Mimics medical (21.0) (Materialise NV, Leuven, Belgium) (Figure 1). The transverse CT images were classified by combining the reconstructed sagittal and coronal positions. A total of 3/5 of the classified data was used for training, 1/5 for testing, and 1/5 for verification. The images were converted from DICOM format to PNG format.

### 2.3. Convolutional Neural Networks

The CNN used in this study includes convolution layer, full connection layer, and pooling layer. The convolutional layer is the basic structure of convolutional neural network, which can obtain local information of image by acting on local image region with a certain size of convolution kernel [12, 13]. The general form of the convolution layer is shown in the equation (1).

(1) $$\begin{array}{c} x_{j}^{l}=f\left(\underset{k\in M_{j}}{\sum }x_{k}^{l-1}*k_{jk}^{l}+b_{j}^{l}\right). \end{array}$$

The pooling layer is essentially a “down-sampling” operation. Different from the convolutional layer operation, the pooling layer does not contain parameters to be learned. The general expression is as shown in the equation (2).

(2) $$\begin{array}{c} x_{j}^{l}=f\left(\beta_{j}^{l}\text{down}\left(x_{j}^{l-1}\right)+b_{j}^{l}\right). \end{array}$$

The full connection layer is generally located at the end of the network. Two-dimensional vector features obtained from the convolution layer and pooling layer are converted into one-dimensional vectors for classification, and the general expression is shown in the formula (3).

(3) $$\begin{array}{c} x_{j}^{l}=f\left(w^{l}x^{l-1}+b^{l}\right). \end{array}$$

### 2.4. Transfer Learning

The parameter training of CNN requires a large number of training samples; so, this paper adopts transfer learning to solve the problem of insufficient training samples [14]. Transfer learning can solve the problem of learning small sample data with existing knowledge, thus improving the classification accuracy of small sample data sets by CNN [15]. Compared with traditional machine learning methods, transfer learning no longer needs enough and available training samples to obtain a good classification model nor does it require that the training samples and the new test samples used for learning meet independent homodistribution [16, 17].

In this study, based on the transfer learning strategy, the convolutional neural network is trained as a pretraining model. The weight parameters of the pretraining model are transferred to the training model. Finally, various parameters are fine-tuned and optimized, the whole network is trained on the training set to update the parameters, and finally, the new model weight is obtained. The specific process is shown in Figure 2.

### 2.5. Model Training and Validation

CNN trains the model, including image format conversion, random classification, training, and testing. The specific training diagram is shown in Figure 3. The genetic algorithm (GA) was used to optimize the parameters [18, 19]. To verify the optimized parameters, the optimized parameters after training were printed once, and the damaged area of the model was observed for comparison.

### 2.6. Operation Method

The optimized parameters were used to build a 3D model, and the aortic arch model was printed in 3D entity (Figure 4). After diagnosis and evaluation of the surgical indications in assistance of the 3D models, we run simplified Sun's procedure under hypothermic cardiopulmonary bypass with selective antegrade cerebral perfusion on all 3 patients. The procedure of the surgery is briefly illustrated in Figure 4(d).

## 3. Results

### 3.1. 3D Reconstruction Printing and Surgical Results

Three-dimensional reconstruction model of aortic arch tends to theoretical model (Figure 1(e)). The damaged area of the model printed with optimized parameters was 0.021 mm^2^ (mean), which was not significantly different from the theoretical value (mean 0.023 mm^2^). In addition, simplified Sun's procedure was applied as planned on each of the 3 patients, and the relevant information are also listed in Table 1. The aortic arch is replaced, a stented elephant trunk is implanted, the autologous brachiocephalic vessels are preserved, and the left subclavian artery is anastomosed to the left common carotid artery.

### 3.2. Postoperative Follow-Up Results

The intraoperative findings of the aortic arch were all consistent with the reconstructed models. Of these three patients, one patient (patient 1 in Table 1) died due to multiple organ failure and septic shock on the 11th day after surgery. The other 2 patients were cured, no reoperation was reported, and their cardiac functions were both defined as class I during the 13 and 20 months of follow-up, respectively.

## 4. Discussion

As one of the treatments for aortic dissection aiming at reconstruction of the aortic arch, simplified Sun's procedure has the similar cardiopulmonary bypass time, selective antegrade cerebral perfusion time, and short-time outcomes with that of conventional Sun's procedure [6]. The advantage of this simplified procedure is that it preserves the autologous brachiocephalic vessels of the patients, leading to a high long-term patency rate. In addition, the reduced anastomoses simplify the operation and reduce the related complications. What is more, the anastomosis of the aortic arch is applied between the left common carotid artery and the left subclavian artery in this procedure, and the relatively clear visualization of the anastomotic site combined with limited separation of the arch makes it more facilitated to do anastomosis. In this study, for the patient who died after surgery, the cause of death was not related to either the preservation of brachiocephalic vessels or the arch anastomosis in the surgery. This patient had a long-term history of smoking. Therefore, it was difficult to control his postoperative pulmonary infection, which led to his multiple organ failure and septic shock.

Aortic dissection occurs and progresses rapidly, leaving a small window of time for clear diagnosis and development of a surgical plan. The diagnosis and the evaluation of surgical indications require precise understanding of the details of the aortic arch and the brachiocephalic vessels, as well as the openings of the branched vessels. Considering the limited cases and relatively fewer training of surgeons in low-volume heart centers like ours, the preoperative surgical plan is particularly important for the application of such a complicated surgery. Preoperative aortic CTA examination is essential for the diagnosis of Stanford type A dissection and is also the fundamental basis for determining the preservation of autologous brachiocephalic vessels [20]. However, the flat image of CTA cannot fully satisfy us with enough details. In some patients with type A aortic dissection, before surgery, according to the CTA image, we planned to preserve the autologous brachiocephalic vessels, but it revealed that the opening of the vessels was slightly involved in the dissection during operation. In that situation, we had to perform conventional Sun's procedure instead of the simplified one, and the change of surgical procedure could increase the risk of surgery [21].

Compared with reconstructed CTA images on the screen, 3D printing models can be more helpful, since it allows us to intuitively view the entire internal conditions of the affected aortic arch and the branched vessels and let us better define the specific condition of the aortic lesions [22, 23]. Precision medicine is an important direction of future medical development. In this paper, CNN is used to train CT images. Transfer learning is applied to model training to solve the problem of small sample size. The GA was used to optimize, and the corresponding manufacturing parameters were obtained [24]. In our study, the model of 3D reconstruction based on image features extracted by the CNN algorithm is closer to the theoretical value. Therefore, it makes it possible for us to develop a surgical plan accurately and even to simulate the surgical procedure. As in this study, the intraoperative findings were all consistent with that of the reconstructed models of the patients; therefore, we could run these surgeries exactly as planned. In addition, two cured patients were followed up for 13 months. No reoperation was performed, and all patients had grade I cardiac function. Li et al. showed that the total endovascular repair for false lumen stent-graft implantation was feasible and minimally invasive [25], and the postoperative recovery of patient is similar to that of our patients.

After obtaining the CTA data, 3D reconstruction of images and model printing can be done within 6 hours; so, we do not need extra time, since it can be done simultaneously with preparation of the operation before surgery. The cost of 3D printing is about $ 150 per person, that is affordable to most of the patient, and it is free of charge in this study.

There are several limitations to our study. Given the small sample size and short follow-up time in this study, more information should be gained with more patients and longer time of follow-up in the future. In addition, the algorithm is too long, affecting the calculation time.

## 5. Conclusion

In summary, the application of 3D printing models based on the CNN is feasible and can be benefit to low-volume heart centers in performing Sun's procedure with preservation of autologous brachiocephalic vessels.

## Figures and Tables

**Figure 1:** 3D reconstruction process diagram based on CNN model feature extraction. Coronal plane (a), horizontal plane (b), and sagittal plane (c). (d) CNN radiomic feature extraction. (e) 3D reconstruction model of the aortic arch.

**Figure 2:** Illustration of model fine-tuning.

**Figure 3:** The workflow of model training.

**Figure 4:** Preservation of autologous brachiocephalic vessels in the treatment for Stanford type A aortic dissection with assistance of three-dimensional (3D) printing. (a) Bottom view of the aortic arch in 3D image, no sign of dissection, or hematoma around the opening of the brachiocephalic vessels and the vessels themselves. (b) 3D printing model of the aortic arch (bottom view). (c) 3D printing model of the aortic arch (anterosuperior view). (d) Illustration of the surgical procedure, the aortic arch is replaced, a stented elephant trunk is implanted, the autologous brachiocephalic vessels are preserved, and the left subclavian artery is anastomosed to the left common carotid artery.

**Table 1:** Clinical data of patients.

	Patient 1	Patient 2	Patient 3
Age (years)	67	54	48
Gender	Male	Male	Male
Hypertension	Yes	Yes	Yes
Initial symptom	Chest pain	Chest tightness	Chest pain
Time from onset to hospitalization (days)	1	3	1
CPB time (mins)	133	167	179
Aortic crossclamping time (mins)	64	82	99
SACP time (mins)	21	24	24
Concomitant procedure	Ascending aorta replacement	Bentall procedure	Bentall procedure

CPB: cardiopulmonary bypass; SACP: selective antegrade cerebral perfusion.

## Data Availability

The data used to support the findings of this study are available from the corresponding author upon request.
